RETRACTED

# Up-regulated circular RNA VANGL1 contributes to progression of non-small cell lung cancer through inhibition of miR-195 and activation of Bcl-2

**DOI:** 10.1042/BSR20182433

**Published:** 2019-06-04

**Authors:** Liuxin Wang, Huiping Ma, Weixiang Kong, Bing Liu, Xueqing Zhang

**Affiliations:** Department of Respiration, Jining No.1 People’s Hospital, Jining City, China

**Keywords:** apoptosis, Bcl-2, circular RNA VANGL1, microRNA-195, non-small cell lung cancer

## Abstract

Circular RNAs (circRNAs), a group of non-coding RNAs, play an important role in cancer biology, and in the present study, we aimed to clarify the expression profiles and biological functions of circRNA circVANGL1 in non-small cell lung cancer (NSCLC). The results showed that circVANGL1 was overexpressed in human NSCLC tissues and cell lines. circVANGL1 expression was closely associated with tumor size, TNM stage and overall survival of NSCLC patients. Further loss-of-function analysis revealed that knockdown of circVANGL1 inhibited proliferation and induced apoptosis in NSCLC cell lines. The migration and invasion of NSCLC cells were also suppressed by circVANGL1 knockdown. In addition, we predicted that circVANGL1 might serve as a competing endogenous RNA (ceRNA), becoming a sink for miR-195, thereby modulating the expression of Bcl-2 in NSCLC cells. Rescue experiments demonstrated that miR-195 inhibitor abrogated the beneficial role of circVANGL1 knockdown in NSCLC cells. Taken together, we conclude that circVANGL1 functions as an oncogene to promote NSCLC progression partly through miR-195/Bcl-2 axis, which might be a novel therapeutic target for NSCLC patients.

## Introduction

Lung cancer is the most commonly occurring cancer around the world. Non-small cell lung cancer (NSCLC), accounting for 85% of all cases, is the most prevalent histological type of lung cancer [1]. Although great achievements have been made in surgical therapy, chemotherapy and molecular targeting therapy, the prognosis of NSCLC patients remains largely dismal. Patients with advanced NSCLC have an average 5-year survival rate of approximately 15% [2]. Therefore, it is worthy and important for us to further identify genetic regulatory networks involved in NSCLC progression.

Circular RNAs (circRNAs), a novel group of endogenous non-coding RNAs, are featured by their covalently closed loop structures without a 5′ cap or a 3′ Poly A tail [3]. circRNAs are widely expressed in mammals with cell-type, tissue and developmental phase-specific manner [4]. It is well documented that many circRNAs play a pivotal role in the initiation and progression of human diseases, especially in cancers [5]. Recently, a novel circRNA, termed as circVANGL1, was identified as an oncogene in bladder cancer [6]. In the present study, we aimed to clarify the expression profiles and biological functions of circRNA circVANGL1 in NSCLC. We believe that our findings might provide new strategies for diagnosis and treatment against this fatal malignancy.

RETRACTED

## Materials and methods

### Tissue specimens

Ninety-five pairs of NSCLC tissues and the matched adjacent normal tissues were collected from patients who had undergone surgical resection at Jining No.1 People’s Hospital (Jining, China). The clinicopathological information of the patients was recorded and listed in Table 1. None of the patients had undergone chemotherapy or radiotherapy prior to surgery. All tissue samples were immediately frozen in liquid nitrogen following surgery and stored at −80 °C for further use. The present study had received approval from the Ethics Committee of Jining No.1 People’s Hospital, and performed in accordance with the World Medical Association Declaration of Helsinki. Written informed consent was obtained from all the subjects.

**Table 1:** Correlation between circVANGL1 expression and clinicopathological characteristics of NSCLC patients

Characteristics	Total number (*n*=95)	circVANGL1 expression		*P*-value
		Low (*n*=46)	High (*n*=49)	
Age (years)				0.267
≤65	44	24	20	
>65	51	22	29	
Gender				0.648
Male	58	27	31	
Female	37	19	18	
Tumor size (cm)				0.028
≤5	64	36	28	
>5	31	10	21	
Histological type				0.619
Adenocarcinoma	50	23	27	
Squamous	45	23	22	
TNM stage				0.019
I-II	61	35	26	
III-IV	34	11	23	
Lymph nodes metastasis				0.105
Yes	39	15	24	
No	56	31	25	

### Cell culture and transfection

Four NSCLC cell lines (A549, H1299, H1975, SPC-A1 and SK-MES-1) and a normal human bronchial epithelial cell line (16HBE), obtained from the Cell Center of Shanghai Institutes for Biological Sciences, were cultured in Dulbecco’s modified Eagle’s medium (DMEM; Invitrogen, Carlsbad, CA, U.S.A.) or RPMI 1640 medium (HyClone, Logan, UT, U.S.A.) supplemented with 10% fetal bovine serum (FBS; HyClone), 100 U/ml penicillin and 100 μg/ml streptomycin in an incubator at 37°C in a 5% CO_2_ atmosphere.

The small interfering RNA (siRNA) targeting circVANGL1 (si-circVANGL1) and the negative control siRNA (si-NC) were synthesized by Guangzhou RiboBio Co., Ltd. (Guangzhou, China). miR-195 mimics, miR-195 inhibitor and the scrambled oligonucleotides (NC) were purchased from Shanghai GenePharma Co., Ltd. (Shanghai, China). Cells cultured on six-well plate were transfected with the oligonucleotides using Lipofectamine 2000 (Invitrogen). After 48 h, the cells were harvested, and transfection efficiency was determined by RT-qPCR analysis.

RETRACTED

### RNA extraction and RT-qPCR analysis

Total RNA was isolated from tissues and cell lines using TRIzol reagent (Invitrogen). Complementary DNA was synthesized using the PrimeScript™ RT reagent kit (TaKaRa, Dalian, China). Thereafter, the RT products were used as templates for PCR amplification using a SYBR® Premix Ex Taq™ II (TaKaRa) on an iCycler iQ™ Real-Time PCR Detection System (Bio-Rad Laboratories, Hercules, CA, U.S.A.). The relative expression levels of circVANGL1 and miR-195 were calculated using the 2^−ΔΔ*C*^_t_ method [7]. Glyceraldehyde-3-phosphate dehydrogenase (GAPDH) or U6 snRNA was used as an internal reference.

### MTT assay

Cells were seeded into each well of a 96-well plate (5 × 10^3^ cells/well), and cell proliferation was determined by 3-(4,5-dimethylthiazol-2-yl)-2,5-diphenyl-2H-tetrazoliumbromide (MTT) assay. At indicated time points, we added 20 μl of MTT reagent (0.5 mg/ml; Merck KGaA, Darmstadt, Germany) to each well. Cells were then incubated at 37°C for additional 4 h. After the supernatants were removed, DMSO (150 μl) was added to each well, and the plates were shaken for 10 min to dissolve the crystals. The optical density (OD) value of each well was determined at 490 nm on a microplate reader (MultiskanEX, Lab systems, Helsinki, Finland).

### Cell apoptosis analysis

Cell apoptosis was detected using the Annexin V-FITC Apoptosis Detection Kit (Beyotime, Shanghai, China). Cells were harvested 48 h after transfection, and stained with 5 µl of Annexin V-FITC and 10 µl of propidium iodide (PI) in the dark for 15 min at room temperature. Stained cells were subjected to a flow cytometer (BD Biosciences, Franklin Lakes, NJ, U.S.A.). Data were analyzed using Cellquest Pro software (BD Biosciences).

### Transwell assay

Cell migration and invasion assays were performed using transwell chambers (Corning Inc., Corning, NY, U.S.A.) using 8-μm sized pore membrane coated with matrigel (for invasion assay) or without matrigel (for migration assay). Cells in serum-free medium were placed into the upper chamber, and 500 μl medium containing 10% FBS was added to the lower chamber. Following incubation for 48 h, the cells remaining on the upper membrane surface were removed, whereas the cells that passed through the pores were fixed with 4% paraformaldehyde and stained with 0.1% Crystal Violet. The number of migrated or invaded cells was counted randomly in five fields of each membrane.

### Western blot analysis

The total protein of samples was extracted using RIPA lysis buffer (Beyotime). Identical quantities of proteins were separated by SDS/PAGE gel, and transferred to PVDF membranes (Millipore, Bedford, MA, U.S.A.). The membranes were blocked with 5% non-fat milk for 2 h, and probed with primary antibodies at 4°C overnight. Afterward, PVDF membranes were incubated with the specific HRP–conjugated secondary antibodies for 1 h at room temperature. Immunoreactive bands were detected by using the Immobilon ECL substrate kit (Millipore), and quantitated by ImageJ 3.0 software (http://imagej.nih.gov/ij/). GAPDH was used as the internal reference.

RETRACTED

### Dual-luciferase reporter assay

The fragment of circVANGL1 or the 3′-UTR of Bcl-2 containing predicted miR-195 binding site was subcloned and inserted into the psiCHECK-2 vector (Promega, Madison, WI, U.S.A.). The binding sites were mutated using the GeneTailor™ Site-Directed Mutagenesis System (Invitrogen). HEK293T cells were seeded into 24-well plates and co-transfected with luciferase reporter vector and miR-195 mimics or NC. The luciferase signals were measured 48 h after transfection using the Dual-Luciferase Reporter Assay System (Promega).

### Statistical analysis

All statistical analyses were performed using GraphPad Prism 6.0 software (GraphPad Software, San Diego, CA, U.S.A.) and SPSS 18.0 software (SPSS Inc., Chicago, IL, U.S.A.). Experimental data were expressed as mean ± standard deviation (SD), and the differences between groups were analyzed using Student’s *t* test or one-way ANOVA. The correlation between circVANGL1 expression and clinicopathological characteristics of NSCLC patients was evaluated using chi-square test. Survival curves were generated using the Kaplan–Meier method and assessed with the log-rank test. A value of *P*<0.05 was considered to indicate a statistically significant difference.

## Results

### circVANGL1 is overexpressed in NSCLC

To investigate the potential role of circVANGL1 in NSCLC, we first performed RT-qPCR analysis to determine the circVANGL1 expression in human NSCLC tissues and cell lines. As shown in Figure 1A, the expression of circVANGL1 in NSCLC tissues was remarkably higher than that of adjacent normal tissues. Similarly, circVANGL1 expression levels were also significantly higher in NSCLC cell lines (A549, H1299, H1975, SPC-A1 and SK-MES-1) than that in the normal human bronchial epithelial cell line (16HBE) (Figure 1B).

**Figure 1:** circVANGL1 is overexpressed in NSCLC (**A**) RT-qPCR analysis of circVANGL1 expression levels in NSCLC and paired adjacent normal tissues from 95 patients. (**B**) RT-qPCR analysis of circVANGL1 expression levels in NSCLC cell lines and normal 16HBE cells. The data are shown as mean ± SD from three independent experiments *in vitro*. *P<0.05 vs. 16HBE cells. (**C**) Kaplan–Meier analysis of the association between circVANGL1 expression and overall survival in NSCLC patients.

RETRACTED

The mean value of circVANGL1 expression in NSCLC tissues was chosen as the cut-off point for allocating 95 NSCLC patients to low expression group (*n*=46) and high expression group (*n*=49). We found that circVANGL1 expression was closely associated with tumor size (*P*=0.028) and TNM stage (*P*=0.019) of NSCLC patients (Table 1). Furthermore, Kaplan–Meier survival analysis revealed that high circVANGL1 expression was also associated with unfavorable overall survival of NSCLC patients (Figure 1C).

### circVANGL1 knockdown induces NSCLC cell apoptosis

We then selected A549 and H1299 cells with relatively high circVANGL1 expression for further experimental analysis. To investigate the biological functions of circVANGL1 in NSCLC cells, we used RNA interference to knock down the expression of circVANGL1 in these two cells. The transfection efficiency was verified by RT-qPCR analysis (Figure 2A). Moreover, we assessed cell proliferation by MTT assay and found that knockdown of circVANGL1 significantly suppressed the proliferation of A549 and H1299 cells (Figure 2B). Besides, as determined by flow cytometric analysis, circVANGL1 knockdown in A549 and H1299 cells significantly increased the percentage of apoptotic cells (Figure 2C). In addition, Western blot analysis confirmed that circVANGL1 knockdown increased the expression of pro-apoptotic protein Bax, and decreased the expression of anti-apoptotic protein Bcl-2 in both A549 and H1299 cells (Figure 2D).

**Figure 2:** circVANGL1 knockdown induces NSCLC cell apoptosis (**A**) RT-qPCR analysis of circVANGL1 expression levels in A549 and H1299 cells after transfection. (**B**) The proliferation abilities of A549 and H1299 cells after transfection were determined by MTT assay. (**C**) The apoptotic rates of A549 and H1299 cells after transfection were determined by flow cytometric analysis. (**D**) Western blot analysis of Bax and Bcl-2 protein expression levels in A549 and H1299 cells after transfection. The data are shown as mean ± SD from three independent experiments *in vitro*. *P<0.05 vs. si-NC-transfected cells.

### circVANGL1 knockdown inhibits NSCLC cell migration and invasion

Migration and invasion are two important features of cancer cells. We then performed transwell assay to examine the effects of circVANGL1 on migration and invasion abilities of NSCLC cells. As demonstrated in Figure 3, in A549 and H1299 cells, the numbers of migrated and invaded cells were significantly reduced when circVANGL1 was knocked down.

**Figure 3:** circVANGL1 knockdown inhibits NSCLC cell migration and invasion The migration and invasion abilities of A549 and H1299 cells after transfection were determined by transwell assay. The data are shown as mean ± SD from three independent experiments *in vitro*. *P<0.05 vs. si-NC-transfected cells.

RETRACTED

### circVANGL1 acts as a competing endogenous RNA of miR-195 in NSCLC

We then explored whether circVANGL1 could act as a competing endogenous RNA (ceRNA) of miRNAs in NSCLC, and through the Starbase database (http://starbase.sysu.edu.cn/index.php), the potential binding sites of miR-195 were identified in the circVANGL1 sequence (Figure 4A). To confirm the above prediction, dual-luciferase reporter assay was then performed, and the results demonstrated that co-transfection with miR-195 mimics and circVANGL1-WT resulted in significantly decreased luciferase activity in HEK293T cells (Figure 4B). In addition, as shown in Figure 4C, circVANGL1 knockdown notably increased miR-195 expression levels in A549 and H1299 cells. We also observed that miR-195 was down-regulated in NSCLC tissues (Figure 4D), and the expression of circVANGL1 had the adverse correlation with miR-195 in NSCLC tissues (r = −0.226, *P*=0.028; Figure 4E).

**Figure 4:** circVANGL1 acts as a ceRNA of miR-195 in NSCLC (**A**) Putative miR-195 binding sequence in circVANGL1 fragment. (**B**) The luciferase activity of circVANGL1-WT or circVANGL1-MUT in HEK293T cells after transfection with miR-195 mimics or NC. (**C**) RT-qPCR analysis of miR-195 expression levels in A549 and H1299 cells after transfection. The data are shown as mean ± SD from three independent experiments *in vitro*. *P<0.05 vs. NC or si-NC-transfected cells. (**D**) RT-qPCR analysis of miR-195 expression levels in NSCLC and paired adjacent normal tissues from 95 patients. (**E**) The correlation between circVANGL1 and miR-195 expression in NSCLC tissues.

### miR-195 targets Bcl-2 in NSCLC

Next, we used TargetScan (http://www.targetscan.org/vert_71/) to identify the target genes of miR-195, and found that the 3′-UTR of Bcl-2 matched the seed sequence of miR-195 (Figure 5A). In addition, a significant decrease in luciferase activity was observed in HEK293T cells co-transfected with Bcl-2-WT and miR-195 mimics (Figure 5B). Moreover, we found that miR-195 overexpression decreased the protein expression levels of Bcl-2 in A549 and H1299 cells (Figure 5C).

**Figure 5:** miR-195 targets Bcl-2 in NSCLC (**A**) Putative miR-195 binding sequence in the 3′-UTR of Bcl-2 mRNA. (**B**) The luciferase activity of Bcl-2-WT or Bcl-2-MUT in HEK293T cells after transfection with miR-195 mimics or NC. (**C**) Western blot analysis of Bcl-2 protein expression levels in A549 and H1299 cells after transfection. The data are shown as mean ± SD from three independent experiments *in vitro*. *P<0.05 vs. NC-transfected cells.

RETRACTED

### miR-195 inhibitor blocks the effects of circVANGL1 knockdown in NSCLC cells

We subsequently performed rescue experiments to verify whether the effects of circVANGL1 on NSCLC cell apoptosis were partly mediated by regulation of miR-195/Bcl-2 axis. As shown in Figure 6A, co-transfection with miR-195 inhibitor rescued the increased Bax expression and decreased Bcl-2 expression in A549 and H1299 cells with circVANGL1 knockdown. Moreover, the increased apoptosis rates in si-circVANGL1-transfected A549 and H1299 cells were remarkably diminished by miR-195 inhibitor (Figure 6B).

**Figure 6:** miR-195 inhibitor blocks the effects of circVANGL1 knockdown in NSCLC cells (**A**) Western blot analysis of Bax and Bcl-2 protein expression levels in A549 and H1299 cells after transfection. (**B**) The apoptotic rates of A549 and H1299 cells after transfection were determined by flow cytometric analysis. The data are shown as mean ± SD from three independent experiments *in vitro*. *P<0.05 vs. si-NC+NC-transfected cells, ^#^*P*<0.05 vs. si-circVANGL1+NC-transfected cells.

## Discussion

NSCLC is a complex and heterogeneous disease, and its underlying mechanisms remain largely undiscovered and poorly elucidated. circRNAs were previously considered as splicing error by-products, but in recent years, circRNAs have attracted extensive attention owing to their frequent participation in a wide range of biological processes, and their dysregulation often leads to human diseases, including cancers [8]. In lung cancer, a large number of differentially expressed circRNAs have been already identified and are regarded as potential biomarkers [9].

In the present study, we tested the expression of circVANGL1 in NSCLC tissues and cell lines. We also explored the functional role of circVANGL1 in NSCLC cells by applying loss-of-function approaches. The results showed a dramatic increase in circVANGL1 expression not only in NSCLC tissues but also in NSCLC cell lines, suggesting its oncogenic effect. *In vitro* functional assays further showed that circVANGL1 knockdown suppressed the malignant traits of NSCLC cells, including proliferation, migration and invasion. Apoptosis is often regulated by Bcl-2 family, including Bcl-2 and Bax [10], and this study also showed that circVANGL1 knockdown promoted cell apoptosis, decreased Bcl-2 expression and increased Bax expression in NSCLC cells.

MiRNAs are another critical class of non-coding RNAs, which exert their biological functions mainly by regulating their downstream targets [11]. Recently, a novel regulatory mechanism has been identified, in which circRNAs can function as ceRNAs to compete together with miRNAs, thereby leading to a loss of miRNA function [12,13]. To investigate the miRNA-related role of circVANGL1, through bioinformatics prediction, we chose miR-195, a well-known tumor suppressor in NSCLC [14,15], as a model miRNA for further analysis, and the binding relationship between circVANGL1 and miR-195 were further proved by the experimental validation. Consistent with the findings in colorectal cancer [16], our results also verified that Bcl-2 was a direct target of miR-195 in NSCLC. Moreover, rescue experiments validated that the effects of circVANGL1 on NSCLC cell apoptosis were partly mediated by regulation of miR-195/Bcl-2 axis.

RETRACTED

In conclusion, for the first time, the present study revealed a novel regulatory mechanism that circVANGL1/miR-195/Bcl-2 axis regulates NSCLC progression, providing a new insight for the development of circRNA-directed diagnostics and therapeutics against this deadly malignancy.

## Abbreviations

Bcl-2: B-cell lymphoma-2
ceRNA: competing endogenous RNA
circRNA: circular RNA
FBS: fetal bovine serum
GAPDH: glyceraldehyde-3-phosphate dehydrogenase
HRP: Horseradish Peroxidase
MTT: 3-(4,5-dimethylthiazol-2-yl)-2,5-diphenyl-2H-tetrazoliumbromide
NSCLC: non-small cell lung cancer
PVDF: poly(vinylidene fluoride)
RIPA: Radio-Immunoprecipitation Assay
RPMI-1640: Roswell Park Memorial Institute-1640
RT-qPCR: Real-time Quantitative polymerase chain reaction
siRNA: small interfering RNA
TNM: Tumor Node Metastasis
VANGL1: Recombinant Vang Like Protien1
